The article "Comparison of Upper Limb Muscle Activity among Workers in Large-Herd U.S. and Small-Herd Italian Dairies" was published in 2016. Journal: Front Public Health.

# Comparison of Upper Limb Muscle Activity among Workers in Large-Herd U.S. and Small-Herd Italian Dairies

**DOI:** 10.3389/fpubh.2016.00141

**Published:** 2016-06-30

**Authors:** Federica Masci, Anthony Mixco, Colleen Annika Brents, Lelia Murgia, Claudio Colosio, John Rosecrance

**Affiliations:** ^1^Department of Health Sciences of the University of Milano and the International Centre for Rural Health at San Paolo University Hospital, Milan, Italy; ^2^Department of Environmental and Radiological Health Sciences, Colorado State University, Fort Collins, CO, USA; ^3^Department of Agraria, University of Sassari, Sassari, Italy; ^4^Department of Environmental and Occupational Health, Colorado School of Public Health, Fort Collins, CO, USA

**Keywords:** milking, surface electromyography, ergonomic, dairy work, musculoskeletal disorders

## Abstract

**Objectives:**

Commercial cow milking tasks, regardless of dairy size, have been documented in many regions of the world as strenuous work requiring high muscular effort, awkward positions, and task repetition. Large-herd dairies are common in the U.S., while Europe historically has mostly small-herd dairies. The objective of this study was to compare the upper limb muscle activity during milking tasks between workers at large-herd U.S. dairies and small-herd Italian dairies. This is the first international study directly comparing upper limb muscle activity among dairy workers from different countries using identical methods.

**Methods:**

Data were collected at 6 large-herd dairies in the U.S. region of Colorado and at 21 small-herd Italian dairies in the Lombardy region. Surface electromyography (sEMG) from the trapezius, anterior deltoid, biceps brachii, wrist flexors, and wrist extensors muscles was recorded from all participating workers (*N* = 65). Electromyography data were normalized to functional maximum voluntary contractions. Anthropometric measurements were also recorded.

**Results:**

Upper limb muscle activity was generally greater among workers in the large-herd U.S. dairies compared with small-herd Italian dairies. The amount of muscular rest as a percent of the work time was significantly greater among large-herd U.S. dairy workers.

**Conclusion:**

The differences revealed in sEMG and percent muscular rest among workers from the U.S. and Italy are likely due in part to differences in work processes adopted by fast-paced industrialized large-herd dairies compared with the slower, but sustained work processes performed at small-herd dairies.

## Introduction

The work of milking dairy cows has been performed throughout the world for thousands of years (1). Although farms in some developing countries continue traditional methods of manual hand milking, the majority of the world’s dairy industry has modernized in the past 50 years from vacuum bucket milking to advanced dairy parlor designs (2) that include automation and precision dairy farming systems. According to Schroeder “technology and increased access to data are enabling dairy farmers to make smarter day-to-day decisions to improve cow health, production, and on-farm efficiencies” (3). Many of the same technological and process changes that have driven efficiency on farms have led to less than ideal ergonomic design within the dairy parlor. Poor system and task design can increase the worker’s risk of developing occupationally related musculoskeletal symptoms (MSSs) and musculoskeletal disorders (MSDs).

Occupationally related MSSs and MSDs often develop from work tasks characterized by excessive exposure to work tasks involving forceful muscle exertions, high number of repetitive motions, and awkward body postures (4, 5). Many of today’s milking systems expose the dairy parlor workers to the same risk factors (high muscle loads, repetition, and awkward postures) for MSSs and MSDs (6–10). Regardless of milking stall design, herd size of dairy operation, or geographical region, from an ergonomics perspective, milking tasks have been documented as involving strenuous work with high muscular loads, high repetition and awkward postures on the upper limb (6, 7, 9–12).

Unfortunately, there are very few international studies comparing occupational risk factors and health outcomes related to dairy work between countries. Recently, Kolstrup and Jakob compared the prevalence of MSSs and MSDs between groups of dairy workers from Sweden and Germany (10). International studies comparing upper limb muscle activity of workers performing milking tasks between any two countries have not been reported previously. Although herd sizes are generally larger in U.S. dairies as compared with Italian, both countries predominately use loose housing systems performed in milking parlors (herringbone, parallel, or rotary configurations), which involve very similar milking processes and work tasks.

Due to the consistently high prevalence of injuries among dairy workers globally, it is prudent for researchers to pool resources and expertise to study and address this international occupational challenge. Thus, the objective of this study was to compare the upper limb muscle activity among workers performing milking tasks in large-herd U.S. dairies with workers in small-herd Italian dairies. The research team conducted this study with the same equipment, methods, and data processing techniques at dairies in the U.S. state of Colorado and the Lombardy region of Italy.

### Dairy Industry Status and Profile in U.S.

Dairy production is a significant component of the U.S. economy and is second only to beef among all livestock industries, with about 138,000 people employed annually in the U.S. (13). The dairy workforce force consists predominantly of hired labor, and estimates indicate that 57,000 are foreign born, with the main ethnic demographic being Latino (13, 14). According to the U.S. Department of Agriculture, the dairy sector in 2015 accounted for 43,584 farms and over 9.3 million dairy cows that collectively produced 94.6 million metric tons of milk (15), which make U.S. the second largest world cow milk producer after the European Union.

Among all U.S. dairy operations (family as well as corporate-owned and operated), the mean herd size is 214 cows. Over the last decade, there has been a shift in farm structure from small (<500 cows) to large (1,000–2,000 cows) and mega-herd (2,000+ cows) dairies (16, 17). Approximately half of the total number of milking cows in the U.S. are raised on large farms with at least 1,000 heads, while smaller farms account only for 17% of total animals (18). As herd size increases, dairy operations become remarkably different than the family farm in terms of management and employment practices as well as the organization of work processes (14). The large- and mega-herd dairy operations are highly mechanized, automated, and typically require one worker for every 80–100 cows, excluding the cropping operations. The fast-paced mechanized milking processes at mega-herd dairies require high task specificity with workers focusing on fewer components of the total milking system. USDA statistics for Colorado indicate the presence of 148,000 cows and 120 licensed dairy farms, which produced 1,701 million kilograms of milk (15). The mean herd size in Colorado was 1,233 head indicating a high intensity dairy region (15).

### Dairy Industry Status and Profile in Italy

In Italy, the dairy industry as a whole (production of all dairy products) is the largest food sector contributing more than 12% to the national food sales. The most recent data from 2016 indicates that there are 35,177 dairy operations and 186 millions cows contributing to a total milk production of more than 11,152 million kilograms per year (19). Italian dairy farms are generally characterized by a very small herd size with 53 cows as the national average and with an average farm production of 315,000 kg of milk per year (19). Italian cow milk production is most concentrated in the northern regions of the country (Lombardy, Emilia-Romagna, Veneto, and Piedmont), which account for 65% of the farms, 77% of the cows, and 75% of the total milk production (20, 21). Lombardy is the region with the highest number of dairy farms (17% of the national value), which raise more than one-third of the Italian dairy cows producing 44% of the Italian milk with an average yield over 9,152 kg/year (22, 23). Due to the significant reduction of dairy farms, average herd sizes have almost doubled since the 1990s. However, in 2011, 90% of Italian dairy farms still had less than 100 cows, while the number of operations with at least 1,000 cows was only 14 (23).

Italian dairy farming is still principally based on family managed operations that employ more than 100,000 workers throughout the country (24). Immigrants from India and Pakistan are a significant and growing part of dairy workforce, particularly, in the Lombardy region (25–27). The majority of dairy farms milk cows twice or three times a day, with herringbone and parallel milking parlors the most common.

## Methods and Procedures

### Participants

Six large-herd dairies in the U.S. state of Colorado that had an average dairy herd size of 2,200 head, and 21 small-herd dairies in the Lombardy region of Italy with an average herd size of 350 head participated in the study. A sampling method of convenience rather than randomization was employed. Only subjects aged 18 years or older and free from current musculoskeletal pain at the time of data collection were recruited for participation. An additional eligibility criterion for the Italian sample was not to have had any wrist surgery in the previous 3 years. Participant recruitment was conducted through verbal announcements by supervisors and owners at the dairy and by printed notices posted in the break rooms at the dairies. In the U.S., the research team had working relationships with six dairies, all of who participated. Of the 36 possible parlor workers at these dairies, 28 participated (26 used in data analyses), while the other workers were not available at the data collection time (*N* = 1), not interested (*N* = 6), or met exclusion criteria (*N* = 1). In Italy, 21 out of 40 dairies contacted and agreed to participate in the study. Of the 45 possible parlor workers at these 21 dairies, 40 participated (39 used in data analyses), while the others were not available at data collection time (*N* = 3) or met exclusion criteria (*N* = 2). Subjects in U.S. were compensated $30 in addition to their normal wage for participation, whereas subjects in Italy received their usual wage only. This study was carried out in accordance with the recommendations of Institutional Review Board of the investigator’s universities (Colorado State University and University of Milan) with written informed consent from all subjects. All subjects (including dairy company owners) gave written informed consent in accordance with the Declaration of Helsinki.

### Data Collection Procedures

Anthropometric measurements were recorded from all subjects in both the U.S. and Italian research sites, according to methods described by Rodgers (28) and Mixco et al. (29). These measurements included functional overhead reach, functional standing height (wearing shoes), shoulder acromial height, forward functional reach, and grip breadth, which were measured as the circumference between the thumb and middle finger. In both the countries, surface electromyography (sEMG) with a sampling frequency of 1,000 Hz using Biometrics DataLOG (Biometrics, England) was collected from the upper trapezius, anterior deltoid, biceps brachii, wrist flexors, and wrist extensors as described in detail previously (29). At the U.S. dairy farms, data were recorded for the length of time it took to completely milk a pen of cows (range of 225–275 cows), approximately 45–90 min. At Italian dairies, sEMG was recorded for at least 60 min but not more than 90 min depending on the number of cows to be milked and worker break times.

Functional maximum voluntary contractions (fMVCs) were recorded to normalize sEMG data of each muscle. Prior to the collection of fMVC data, a 30-s baseline resting sEMG signal was recorded from each muscle of each subject, which establishes a minimum resting muscle activity. At least three fMVC trials were conducted for each subject for each muscle group. After each trial, a maximum muscle contraction value was determined using the middle 3 s of the root mean square (RMS) processed sEMG signal.

### Milking Tasks

Workers in the large-herd U.S. and small-herd Italian dairies in this study performed similar milking tasks during the respective data collection periods. All large-herd U.S. dairy workers in this study completed five distinct milking tasks within the dairy parlor. These tasks included (1) pre-dipping (disinfectant solution lifted to or sprayed on the cow teats; see Figure 1), (2) stripping (manually milking teats to stimulate milk production), (3) wiping (cleaning and drying teats with cloth), (4) attaching milking cluster to teats (see Figure 2), and (5) post-dipping (second disinfectant solution lifted to or sprayed on the teats). Ten out of the 21 Italian dairies studied did not perform the pre-dipping or post-dipping tasks as part of normal their milking procedures. Additionally, in 25% of the U.S. and 80% of Italian dairies, workers performed the stripping and wiping tasks together with one upper limb motion. In both the countries, for tasks that could be completed using either the right or left arm, subjects were instructed to use the instrumented arm (hand dominant side). In rotary type parlors, subjects were rotated every 15–20 min through three different process points to conduct the different milking operations (tasks 1–2, 3–4, and 5).

**Figure 1:** **An Italian dairy worker pre-dipping teat in a rotary parlor**.

**Figure 2:** **An American dairy worker attaching milking cluster to cow teats/udder**.

### Muscle Activity Profiles

After normalization of all sEMG data using fMVCs, muscle activity profiles were developed. Temporal analysis of sEMG data was accomplished through standard RMS processing techniques (30). A graphic user interface was created using MATLAB 7.10.0 (Mathworks, Natick, MA, USA) to process sEMG data and obtain mean RMS values. Amplitude probability distribution functions (APDF) was determined for the 10th, 50th, and 90th percentile (31) using custom software (32) developed in LabVIEW (National Instruments, Austin, TX, USA). Percent muscular rest (%MR) of sEMG was determined with a maximum threshold of 0.5% MVC and a minimum gap duration threshold of 0.25 s (33). Another LabVIEW custom software program (32) was used to determine %MR values. Muscle activity profiles were constructed for each muscle with normalized muscle activity expressed as mean RMS, ADPF, and %MR. The muscle activity data were averaged across workers by country to estimate the overall muscle activity and recovery experienced by parlor workers in the U.S. and Italy during the milking tasks.

### Statistical Analysis

This study was a cross-sectional design conducted within the same year in both countries. Statistical analyses were conducted using SAS 9.3 (SAS Institute Inc., Cary, NC, USA). Sample size was determined from power calculations using a conventional alpha level of 0.05, a beta level of 0.20, representing 80% power and effect magnitudes based on previously published EMG data from dairy studies (8, 12). Descriptive statistics for the subjects and muscle activity profiles were computed and summarized. Muscle activity profiles were examined using a random block 2 × 65 × 5 analysis of variance (ANOVA) (dairy location × subject × muscle) with a Tukey Honest Significant difference *post hoc* adjustment to determine differences in the mean RMS, APDF, and %MR variables. Statistically significant interactions between muscle and dairy location (U.S. or Italy) were assessed by examining the simple main effects. Statistically significant differences for anthropometric measures between workers at U.S. and Italian dairies were assessed using Chi squared (χ^2^) test and by examining the likelihood ratio test statistic. Statistical significance was set *a priori* at *p* < 0.05.

## Results

### Participants

A total of 65 workers (26 U.S. and 39 Italy) from 27 dairies (6 U.S. and 21 Italy) participated in the study and had complete data that were used in the analysis of results. All U.S. workers self-identified as Latino with reported countries of origin that included North and Central America (Figure 3). The origin of the Italian workers included the continents of Asia, Africa, Middle East, and Europe (Figure 4). The χ^2^ statistical tests on anthropometric data indicated that the two subject populations were similar in stature but had significant differences in forward functional reach (Table 1). The mean age and work experience of workers employed in the Italian dairies was significantly greater than that of workers in U.S. dairies (Table 1). All, except one (U.S. woman), participants were males. The majority of workers were right-hand dominant; U.S. 97% and Italy 95%.

**Figure 3:** **Distribution of country of origin for the U.S. dairy subjects**.

**Figure 4:** **Distribution of country of origin for the Italian dairy subjects**.

**Table 1:** **Anthropometric data for U.S. large-herd and Italian small-herd dairy workers**.

	U.S. dairy workers mean (SD)	Italian dairy workers mean (SD)	*p* < 0.05
Age (SD)	29.7 (9.80)	43.1 (11.00)	*
Work experience (SD)	3.4 (4.80)	13.4 (10.75)	*
BMI (SD)	26.4 (4.20)	27.34 (3.95)	−
Body mass (SD)	73.9 (16.2)	79.0 (11.19)	−
Functional stature (SD)	166.4 (9.30)	165.0 (35.41)	−
Functional overhead reach (SD)	204.0 (23.18)	204.8 (31.05)	−
Functional forward reach (SD)	61.3 (3.50)	65.5 (4.90)	*
Shoulder height (SD)	140.1 (7.50)	145.1 (5.53)	−
Grip breadth (SD)	15.5 (2.33)	16.1 (1.22)	−

*Statistically significant difference between groups. Mean and (SD) are shown for each characteristic, *N* = 26 for large-herd U.S. workers, *N* = 39 for small-herd Italian workers. Age and work experience in years; body mass in kilograms; functional stature, forward functional overhead reach, functional forward reach, eye level height, shoulder height, waist height, and grip breadth in centimeters.

### Muscle Activity Profiles

Profiles of muscle activity characterizing the normalized mean RMS, APDF at the 10th, 50th, and 90th percentiles and %MR were created for the upper trapezius, anterior deltoid, biceps brachii, wrist flexors, and wrist extensors for both U.S. and Italian dairy workers. As can be seen in Tables 2 and 3, upper limb muscle activity generally was greater among workers in the large-herd U.S. dairies than workers in small-herd Italian dairies. The ANOVA for mean RMS muscle activity indicated a significant interaction (*p* < 0.001) between the dairy size and upper limb muscle when examining the fixed effects. The simple main effects of the interactions (Table 4) revealed significantly greater mean RMS muscle activity for the biceps brachii (*p* < 0.001), upper trapezius (*p* = 0.002), and the wrist flexors (*p* < 0.001) for large-herd U.S. workers than small-herd Italian workers. However, the anterior deltoid (*p* = 0.43) and the wrist extensor (*p* = 0.50) muscles were not significantly different between the two worker groups.

**Table 2:** **Muscle activity profiles by muscle for large-herd U.S. dairies**.

EMG variable	Upper trapezius mean (SD)	Anterior deltoid mean (SD)	Biceps brachii mean (SD)	Wrist flexors mean (SD)	Wrist extensors mean (SD)
10th percentile APDF	1.13 (2.07)	0.15 (0.39)	1.21 (2.22)	0.54 (0.92)	0.40 (0.59)
50th percentile APDF	9.28 (6.61)	3.49 (3.71)	14.58 (11.5)	7.41 (5.10)	9.75 (5.70)
90th percentile APDF	31.44 (21.04)	43.36 (36.26)	51.22 (38.86)	44.11 (31.13)	36.74 (21.40)
Mean RMS (%fMVC)	0.58 (9.19)	9.74 (3.71)	19.44 (13.87)	12.73 (6.24)	14.02 (7.73)
%MR	6.64 (7.24)	22.77 (12.75)	9.45 (7.34)	13.58 (8.25)	13.16 (6.69)

*RMS, root mean square; APDF, amplitude probability distribution function; %fMVC, percent functional maximum voluntary contraction; %MR, percent muscular rest*.

**Table 3:** **Muscle activity profiles by muscle for small-herd Italian dairies**.

EMG variable	Upper trapezius mean (SD)	Anterior deltoid mean (SD)	Biceps brachii mean (SD)	Wrist flexors mean (SD)	Wrist extensors mean (SD)
10th percentile ADPF	0.66 (1.18)	0.16 (0.88)	0.076 (0.69)	0.15 (1.52)	0.23 (1.85)
50th percentile APDF	6.28 (4.29)	3.60 (3.99)	4.38 (2.73)	2.51 (2.67)	9.23 (5.58)
90th percentile APDF	19.50 (12.27)	29.61 (24.31)	19.75 (9.94)	35.85 (48.81)	43.43 (36.76)
Mean RMS (%fMVC)	8.46 (5.35)	8.26 (5.23)	6.86 (4.02)	5.64 (4.12)	14.60 (7.78)
%MR	0.59 (1.22)	4.98 (5.88)	5.36 (10.10)	4.67 (4.55)	5.67 (3.36)

*RMS, root mean square; APDF, amplitude probability distribution function; %fMVC, percent functional maximum voluntary contraction; %MR, percent muscular rest*.

**Table 4:** **Simple main effects of dairy size × muscle interaction from mean RMS muscle activity**.

Muscle	Large-herd U.S. estimated RMS (%fMVC)	Small-herd Italian estimated RMS (%fMVC)	Estimated delta	Adjusted *p*-value
Anterior deltoid	9.62	8.25	1.37	0.42
Upper trapezius	13.47	8.03	5.44	0.002
Biceps brachii	19.32	6.85	12.47	<0.001
Wrist flexors	12.62	5.63	6.99	<0.001
Wrist extensors	13.90	15.06	−1.16	0.50

*RMS, root mean square; %fMVC, percent functional maximum voluntary contraction*.

The upper limb muscle activity expressed at the 50th and 90th percentile of the APDF was also assessed statistically. The ANOVA for the 50th percentile APDF indicated a significant interaction (*p* < 0.001). The simple main effects of these interactions (Figure 5) revealed significant greater activity for the biceps brachii (*p* < 0.001), upper trapezius (*p* = 0.02), and wrist flexors (*p* = 0.0004), but not for the anterior deltoid (*p* = 0.97) and the wrist extensors (*p* = 0.84) when comparing the two worker groups. The results of the 50th percentile APDF analysis were as expected because of the greater intensity and the higher volume of work tasks observed in large-herd U.S. dairy operations versus small-herd Italian dairy milking parlors.

**Figure 5:** **Simple main effects of dairy size × muscle interaction for 50th percentile APDF**. Red line indicates limit values that muscle load should not exceed (31). *p = 0.02, **p = 0.004, and ***p < 0.001. APDF, amplitude probability distribution function.

The ANOVA for the 90th percentile APDF also revealed a significant interaction (*p* < 0.001). For the 90th percentile APDF, the simple main effects of the interactions (Figure 6) revealed significantly greater muscle activity only for the biceps brachii (*p* < 0.001) and not the other upper limb muscles, when comparing large-herd U.S. workers to small-herd Italian workers.

**Figure 6:** **Simple main effects of dairy size × muscle interaction for 90th percentile APDF**. Red line indicates limit values that muscle load should not exceed (31). ***p < 0.001. APDF, amplitude probability distribution function.

The ANOVA for %MR indicated a significant interaction between dairy size and the upper limb muscles assessed (*p* < 0.001). The simple main effects of the interactions indicated that the %MR was significantly greater for the anterior deltoid, upper trapezius, finger flexors, and finger flexors, but not for the biceps brachii (*p* = 0.06) among large-herd U.S. dairy workers relative to small-herd Italian workers. The %MR for all muscles during the working tasks was nearly double for the large-herd U.S. dairy workers as compared with the Italian small-herd dairy workers (Figure 7). These results were not expected as large-herd dairies typically have a higher volume of milking work and a faster work pace compared with small-herd dairies, and therefore, less resting time for workers.

**Figure 7:** **Simple main effects of dairy size × muscle interaction for %MR**. *p = 0.004, **p = 0.002, and ***p < 0.001. %MR, percent muscular rest as percentage of total sEMG recording time.

## Discussion

The primary objective of this investigation was to determine if there were differences in upper limb muscle activity during milking tasks performed by workers in large-herd U.S. dairy operations and workers in small-herd Italian dairies. This objective was accomplished through an analysis of the upper limb muscle activity profiles consisting of the mean RMS, APDF percentiles, and %MR for the upper trapezius, anterior deltoid, biceps brachii, wrist flexors, and wrist extensors for workers in both countries. Based on the previous studies (31) of muscular load, upper limits values have been proposed for preventing excessive muscular load that may contribute to fatigue and injury. The upper limit values for task durations of 1 h or more include: static load levels should not exceed 2% of MVC and must not exceed 5% of MVC; the 50th percentile load level should not exceed 10% of MVC and must not exceed 14% of MVC; and the peak loads (90th percentile) should not exceed 50% of MVC and must not exceed 70% of MVC (31).

The analysis of mean RMS, APDF percentiles, and %MR indicated that the milking activities affected the upper limb muscles differently based on large-herd U.S. workers and small-herd Italian dairy workers. The mean RMS analysis and 50th percentile APDF revealed that among the large-herd dairy workers in Colorado, there was greater intensity of muscle activity for the biceps brachii, upper trapezius, and the wrist flexors. Interestingly, the %MR was significantly greater among workers in the large-herd compared with the small-herd dairy operations. Workers from the large-herd farms had %MR nearly double that of workers on small-herd farms. However, anterior deltoid activity for both mean RMS and 50th percentile APDF were similar between the U.S. and Italian groups. Furthermore, the analyses of %MR revealed that the Italian dairy subjects had less rest for the anterior deltoid muscle. The relative consistency in anthropometrics between the two groups suggests that differences in muscle activity variables may be more related to differences in work methods between the large-herd U.S. and small-herd Italian dairies.

The mean herd size for the Coloradan dairies studied was approximately 2,200 cows, and the mean herd size in Italian dairies studied was 350 cows. In addition, Italian dairies milked their cows twice per day whereas, in the Coloradan dairies, the cows were milked three times per day. The larger herd size and increased frequency of milking in the Colorado dairies results in more cows milked per hour, and thus a faster work pace among milkers was often observed in industrialized milking operations (34). The work pace in the large-herd Colorado dairy parlors was so rapid that the investigators were required to remove all electrodes and equipment from subjects as they were taking a brief rest break between pens of cows. The faster paced high-intensity work in large-herd dairies may partially explain the increased muscle activity recorded among the workers in large-herd U.S. operations in this study. Although muscle activity relative to work pace has not been examined previously within the dairy industry, it has been examined in repetitive assembly work (35). Increasing work pace has been associated with increases, as well decreases, in regard to muscular load during work tasks (35, 36). This suggests that differences in work pace may or may not be related to the differences in muscle activity recorded among large-herd U.S. and small-herd Italian dairy workers.

The most unexpected result of this study was the large amount of %MR recorded among the large-herd U.S. parlor workers, nearly twice as much muscular rest as the smaller-herd Italian dairy parlor workers. This finding was unexpected because of the work pace and workload differences observed between large and small-herd operations. One possible explanation for the significant differences found in %MR between large-herd U.S. and small-herd Italian dairy workers was related to the management of the milking procedures by the dairies studied. All workers tested in the Coloradan dairies performed all five of the milking tasks, pre-dipping, stripping, wiping, attaching, and post-dipping. Work practices at the Italian dairies involved in this study were not as consistent as the U.S. dairies. Ten out of the 21 Italian dairies studied (involving 13 workers) did not perform the pre-dipping or post-dipping tasks as part of their normal milking routine. The definition of %MR requires that muscle activity fall below 0.5% fMVC for at least 0.25 s to be categorized as “rest.” If only three out of five milking tasks were being performed, the task and muscle activity variation in these subjects could be reduced resulting in less muscular rest relative to total task time. Additionally, Italian dairy workers often had brief breaks (up to several minutes) during milking tasks and were required to perform other dairy work activities. These activities included pushing cows into the parlor, hosing off the pit floor and other areas, retrieving supplies, and completing antibiotics injections. Performing a variety of low effort tasks at a slow to moderate pace as in the above activities throughout the data collection period would contribute to the relatively low mean RMS activity and low %MR. In contrast, large-herd U.S. dairy workers performed a set of five tasks that were more repetitive but had rigid tack times that included micro breaks (>0.25 s). It was likely that the repetitive but frequent micro breaks also accounted for some of the increased %MR among the U.S. workers.

An additional procedural difference between U.S. and Italian dairies consisted of the stripping and wiping tasks. In the majority (80%) of Italian dairies, workers performed the stripping and wiping tasks together with the same upper limb motion. This time saving modification of combining two tasks into one further increased the simplification of work allowing the worker to perform tasks at a slower but more continuous pace. It is unlikely that the faster and higher intensity upper limb work observed in large-herd U.S. dairy parlors allows workers to sustain upper limb efforts without adequate rest (micro) breaks built into the work process. Thus, maintaining a healthy dairy workforce free from MSDs may only be possible if workers involved in high intensity repetitive work of the upper limb have adequate %MR.

Other researchers have reported that dairy milking is difficult and physically strenuous work in both large-herd and small-herd operations (7, 9, 10, 37). Additionally, investigators have reported high association between both large-herd and small-herd operations and MSS, MSDs, and workability (6, 9–11, 38–41). This study has clearly demonstrated that there are significant differences in the sEMG of upper limb muscles of large-herd U.S. dairy workers relative to small-herd Italian dairy workers. The differences revealed in sEMG and %MR among workers from Colorado and the Lombardy region are likely due in part to differences in work processes adopted by fast-paced industrialized large-herd dairies compared with the slower, but sustained work of small-herd dairies. Other factors accounting for some of the differences revealed in sEMG and %MR between the groups of workers studied may be related to procedural differences (need for pre-dipping and post-dipping of teats) that may also affect cow health and milk quality.

### Limitations

Many of the limitations in this research were related to the large resources required for international studies of this magnitude. The sampling duration was limited to approximately 1 h per subject. Although the milking tasks are relatively repetitive, this short sampling time may not be representative of the entire shift, especially in Italian dairies where there was greater task variability. Large-herd dairy operations in the U.S. operate 8- to 12-h shifts. Thus, physiologic and muscle fatigue that may be present with full shift work was not measured due to the limited resources. Future research should consider the impact of muscle fatigue by examining full shift data.

The application of sEMG in occupational field studies has limitations due to methodological challenges associated with sEMG recordings. Some of these challenges include variables that can affect the sEMG signal other than the actual muscle activity such as electrode configuration, electrode placement and orientation, procedures for determining a functional MVC, cross talk from other muscles, movement artifact, muscle movement under the surface of the electrode, and tissue impedance and signal processing (30).

## Conclusion

This is the largest multinational study related to the assessment of upper limb muscle activity among dairy workers. This study demonstrated significant differences in the sEMG of upper limb muscles during milking tasks for large-herd U.S. dairy workers relative to small-herd Italian dairy workers. Generally, mean RMS activity of the upper trapezius, biceps brachii, and finger flexors was significantly greater among workers at large-herd U.S. dairies than for workers at small-herd Italian dairies. However, the %MR was significantly greater for the anterior deltoid, upper trapezius, finger flexors, and finger flexors, but not for the biceps brachii among large-herd U.S. dairy workers relative to small-herd Italian dairy workers. The sEMG differences between the two worker groups were likely related to differences in work processes adopted by fast-paced industrialized large-herd dairies compared with the slower, but sustained work processes was performed at small-herd dairies. Other factors accounting for differences revealed in sEMG and %MR between the groups of workers may be related to differences in milking task methods.

## Author Contributions

All authors (FM, AM, CB, LM, CC, and JR) have (1) contributed substantially to the conception or design of the work and/or the acquisition, analysis, or interpretation of the data for the work, (2) participated in drafting the work or revising it critically for important intellectual content, (3) approved the final version to be published, and (4) agreed to be accountable for all aspects of the work in ensuring that questions related to the accuracy or integrity of any part of the work are appropriately investigated and resolved. JR was the local principal investigator and led academic for this part of the grant award. He led the design of the study, providing expertise in sEMG and occupational biomechanics, and made a significant contribution to both the interpretation of data and the writing of the final paper. FM was the doctoral researcher who contributed to study design, led data collection in Italy, contributed to data analysis, and wrote first draft. AM was the doctoral researcher who was involved in the design of the study, led the collection of U.S. data, conducted the data analysis, contributed to interpretation of data, and wrote the first draft. CB was the student researcher contributing to the interpretation of data and co-editing various drafts of the final paper. LM contributed significantly to the conception of the study, developed the manuscript sections on U.S. and Italy dairy profiles, and edited the final manuscript. CC contributed significantly to study conception and design, reviewed manuscripts for the intellectual content and accuracy.

## Conflict of Interest Statement

The authors declare that the research was conducted in the absence of any commercial or financial relationships that could be construed as a potential conflict of interest.
